# Stock Market Reaction to the Announcement of the COVID-19 Lockdown: Evidence from Healthcare Companies in Malaysia

**DOI:** 10.1155/2022/7279233

**Published:** 2022-08-13

**Authors:** Yi Xie, Lingke Zhou

**Affiliations:** ^1^Department of Finance, Faculty of Business, Suzhou Institute of Technology, Jiangsu University of Science and Technology, Zhangjiagang City, Jiangsu Province, China; ^2^Department of Finance and Banking, Faculty of Business and Accountancy, University of Malaya, Kuala Lumpur, Malaysia; ^3^Department of Economics, Faculty of Business, Jiangsu University of Science and Technology, Zhangjiagang City, Jiangsu Province, China

## Abstract

The sudden global pandemic of COVID-19 occurred in Malaysia at the beginning of new 2020, which increased the uncertainty of the economy. As a highly demanded industry during diseases, COVID-19-related news had a mixed influence on investors' confidence in the healthcare industry, so the short-term market reaction of the Malaysian healthcare industry is investigated during this unfolding event. This paper examines whether the “lockdown” suppressed the influence of COVID-19 pandemic on stock performance in 12 listed healthcare companies in Malaysia. We consider the “lockdown” order has different impacts on samples. The hardest hit among the four events is the first announcement of lockdown, whose cumulative average abnormal return (CAAR) is negative (CAAR<0), for its strict movement control. However, the impacts of the following three lockdown events are positive and less severe as the market gradually digest these kinds of news and the deregulation of movement control. Previous studies have justified the influence of disease outbreaks on the stock market; however, this study compensates for other studies by employing the event study methodology (ESM) approach to provide the first empirical evidence of the unprecedented influence of “lockdown” on Malaysian healthcare stock market. This study has practical implications for Malaysian financial markets that the lockdown orders matter for the Malaysian healthcare industry. The empirical results show that the stock market has positively affected the lockdown announcement after the first event. In turn, the policymakers could draw on these results related to stock performance to modify the regulations in the healthcare industry.

## 1. Introduction

It is obvious that the pandemics, such as COVID-19, would influence socioeconomic activities and stock markets worldwide [1–3]. To better control the spread of the pandemic, governments' responses were promoted as lockdown, movement control, and quarantine [4]. COVID-19 pandemic in Malaysia started as a small wave of 22 cases in January 2020 through imported cases, and then, it was followed by an enormous pandemic wave on May 30, 2020, with 7732 confirmed cases and 115 deaths in Malaysia for COVID-19. The World Health Organization (WHO) asserted that the case fatality rate was around 4% and declared a Public Health Emergency of International Concern (PHEIC) due to the rapidly spreading of COVID-19 on January 30, 2020 [5]. All ongoing activities in Malaysia were canceled, and all citizens were under the regulation of the Movement Control Order (MCO). Regarding the Centre for Disease Control and Prevention (CDC), the effective mitigation strategies for reducing the spread of the virus are limiting physical contact between people [6]. Malaysian Minister of Health Dr. Adham Baba announced on March 15, 2020, that Malaysia had 428 cases of newly diagnosed coronary pneumonia, making it the most severe Southeast Asian country under the COVID-19 pandemic wave. Subsequently, on March 16, Prime Minister Muhyiddin Yassin announced the first-phase MCO of Infectious Diseases Act 1988 [7], which was imposed from March 18, 2020.

In conclusion, the Malaysian government has officially announced four MCOs to prevent the spread of this disease in 2020 on March 16, 25, 10, and 23. Malaysian Minister of Health Dr. Adham Baba announced on March 15 that Malaysia had 428 new cases of newly diagnosed coronary pneumonia, making it the most severe Southeast Asian country. Subsequently, on March 16, Prime Minister Muhyiddin Yassin announced the phase 1 MCO of infectious [7] and imposed it from March 18, 2020. Then, phase 2 MCO announced on March 25 that it would be more restricted and extended for another 14 days from April 1 to April 14 in 2020. The phase 3 MCO was announced on April 10, 2020, and would be extended for another fortnight until April 28. Meanwhile, the Malaysian Ministry of International Trade and Industry announced that nine areas would be gradually opened during this period. On April 23, the president announced the implementation of the phase 4 MCO from April 29, 2020, to May 12, 2020.

The healthcare industry, a part of the tertiary industry, offers healthcare services to customers, and the demand for the healthcare sector continued to grow during the COVID-19 pandemic. As Malaysian healthcare business not only depends on the local market but also is a piece of crucial medical equipment exporting industry in which over 90% of the healthcare products manufactured in Malaysia are exported to all parts of the world. This industry gathered more than 200 manufacturers, with nearly MYR14.2 billion investment, meanwhile contributing Malaysia into a global healthcare manufacturing center. It has been announced that the lockdown has obvious potential impacts on supply chain management issues [8], logistics issues [9], exports [10], and production disruptions [11], while the lockdown policies have impacted demand side across different products, and the significant stockpiling of medial items further stimulates its increasing demand [12]. At this stage, this study examines the stock market reaction to the lockdown announcement for the COVID-19 pandemic. For this purpose, the behavior of daily returns before and after these four lockdown announcements made by Prime Minister Muhyiddin Yassin in 2020 has been analyzed. The first research question of this study is “what is the relationship between four lockdown announcements and stock returns in the Malaysian healthcare industry?”. Further, the study also aims to assess the impact of different characteristics of samples in these events. Therefore, we divide the sample by subindustry, asset scale, and firm age to figure out the research question, “what are the different performances of 12 listed healthcare firms in four events?”. To quantify the effects of COVID-19 on Malaysian stock markets of the healthcare industry using ESM to measure the changes in CAR and CAAR to four lockdown events, the traditional event study methodology (ESM) the paper adopts has been widely used for investigating the response of asset prices to new information. However, because the COVID-19 pandemic has become highly topical and is still ongoing, various industries are available with this method. Future studies could use ESM to examine other markets.

The arrangements of the following paper are in these four sections: Section 2 is the literature review of relevant research, Section 3 includes the data and methodology, followed by the empirical results in Section 4, and Section 5 includes the conclusion and implication.

## 2. Literature Review

Baker et al. [13] argue that no infectious disease outbreaks like COVID-19 had such a powerful influence on the stock market. However, little literature has focused on how this pandemic affects the stock market. To summarize the studies on this global disease outbreak, existing literature pays more attention to illness-associated costs of medical or macroeconomic effects arising from morbidity and mortality. Al-Awadhi et al. [14] evaluated the impact of contagious infectious diseases on the stock market across all companies in China, with daily growth in total confirmed cases and in death cases caused by COVID-19. They noted that this disease interacts negatively impacted Chinese stock market returns. Moreover, the results of Baig et al. [15] show that the number of confirmed cases and deaths in the COVID-19 pandemic has a significant negative correlation with the liquidity and volatility of the U.S. equity stock market.

Furthermore, concerning event studies, Carter et al. [16] examined the effects of the COVID-19 outbreak on the stock performance of airline, hotel, and tourism industries in the United States, including 18 airlines, 18 hotels, resorts, and cruise line firms, and 39 restaurants. Their results suggest that larger firms were associated with less negative returns during the COVID-19 outbreak, while firms with greater leverage were penalized more. Chen et al. [17] and Aslam et al. [18] focus on the markets' long-term and short-term stock performance. Their findings supported the time-varying co-integration relationship in the total stock price index and stoking fears of a global pandemic. Liu [19] employs the EGARCH approach to examine the Chinese stock market and finds that the COVID-19 pandemic negatively influences China's composite index, but it varies by different sectors. Chong, Li, and Yip [20] investigate the impact of COVID-19 on the economic figures among cross-countries.

In addition, Fama [21] claims that event study methodology (ESM) explains how quickly asset prices respond to new information. This methodology was proposed by financial experts Fama, Fisher, Jensen, and Roll (FFJR) (1969), while it has been widely used in other areas, such as accounting [22,23], management [24,25], and economics [26,27]. Concerning the literature about the impact factors of abnormal stock returns in the context of ESM, Fama and French [28] empirically explore the items that can affect the abnormal returns of stocks, which are the factors grouped according to the ratio of market capital and book market value of stocks. Renmin [29] proposed the capital asset pricing model to obtain abnormal returns on M&A and studied the market value of listed companies, net asset and operating cash flow of listed companies, and the impact of net profits on abnormal returns. He claims that net assets and market value significantly impact abnormal returns, while other variables fail the test. He et al. (2020) examine the impact of the COVID-19 outbreak on the Chinese stock market. Moreover, they found that the abnormal returns of listed companies on the Shanghai Stock Exchange decreased significantly, whereas the Shenzhen Stock Exchange showed the opposite results. The results show that the COVID-19 pandemic not only hits the traditional industries of China negatively but also creates opportunities for developing high-tech industries. In addition, Wang, Yang, and Li [30] found that the government response to the QE policy alleviated the influence of the COVID-19 pandemic on the Chinese energy market. This study rests on the uncertainty theory [31], which claims that investors will become worried and adopt indiscriminate selling to avoid any future losses in moments of uncertainty. This paper contributes to the limited literature by providing the first empirical evidence on the unprecedented impact of lockdown announcements on the Malaysian healthcare stock market.

## 3. Data and Methodology

### 3.1. Data

The sample selected in this article is listed healthcare industry companies in Bursa Malaysia. The database we used for this study is FTSE Bursa Malaysia KLCI (FBMKLCI). The data of daily stock prices and daily market indices cover the period of May 24, 2019, to May 22, 2020, and the sampling frame of the research is taken from Thomson Reuters Database. There are a total of 13 listed companies in the healthcare industry. We dropped Adventa Berhad in our sample for eliminating illiquid firms because it was suspended for 33 trading days within the sample period. Finally, 12 listed companies are identified from the database in this research, which is listed in Table 1. 

### 3.2. Methodology

This study employs the event study methodology (ESM), which has been widely used to examine the impact of economic or political events on the market reaction and run the data with Stata 15.1 software to assess the effects of four lockdown announcements on the healthcare industry at different periods prior and after the introduction of lockdowns in Malaysia. The selection of the event day is in line with the official media announcements and reports on the Malaysian Ministry of Foreign Affairs website. To ensure that the impacts of the four events are fully reacted within one week, inclusive of the events, the event window in this paper is selected as three trading days before and after every event for (−3, 3). Considering the event may occur on a non-trading day, any event occurs on a non-trading day, we select its next first trading day to study. According to Peterson [32], the estimate window for the model based on daily return is generally between 100 and 300 days, and this study selects 200 trading days before the event to make sure the data are more reliable, and to prevent event windows from overlapping, we select 60 trading days before every event to make sure the stability of the regression coefficients, which lead to the estimation window as (−200, −60).

There are three valuation models for the regular return. Brenner [33] believes that the market model is the most common method of predicting the rate of return, and the predictive power of this model is as good as other complex models. This paper decides to apply the market model (MM) to calculate the returns of 12 listed companies in the Malaysian healthcare industry during the event window. The OLS model is as follows:

(1) $$\begin{array}{c} R_{i,t}=\alpha_{i}+\beta_{i}R_{m,t}+{ɛ}_{i,t}, \end{array}$$

where *R*_*i*,*t*_is the return of the healthcare stock *i* on trading day t:

(2) $$\begin{array}{c} R_{i,t}=\ln\left(P_{i,t}\right)-\ln\left(P_{i,t}-1\right), \end{array}$$

where *R*_*m*,*i*_ is the market return rate on trading day *t*, *β*_*i*_is the covariance of market returns and stock returns on the trading day of stock *i*, *α*_*i*_ is the constant term of stock *i*, and *P*_*i*,*t*_ is the closing price of stock *i* on trading day *t*, that is, the logarithmic value of the closing price of the stock *i* on trading day *t* minus the logarithmic value of the closing price on trading day t-1. Then, we proposed the estimated coefficients from equation (1) to calculate *ɛ*_*i*,*t*_of healthcare stocks.

(1) *Calculation of Abnormal Return (AR)*. The abnormal rate of return is the actual return calculated in Eqs. (1) and (2) minus the normal rate of return, calculated as follows:

(3) $$\begin{array}{c} AR_{i,t}=R_{i,t}-\left({\hat{\alpha }}_{i}+{\hat{\beta }}_{i}R_{m,t}\right), \end{array}$$

where $A{\hat{R}}_{i,t}$ is the abnormal return, *R*_*i*,*t*_ is the normal return of stock *i* stock in period *t* of the event window in Eq. (2), and ${\hat{R}}_{i,t}$ is the normal return evaluated by the market model. After calculating the AR of each sample, the average abnormal return rate (AAR) is calculated as follows:

(4) $$\begin{array}{c} AAR_{t}=\frac{1}{Ν}\sum_{i=1}^{N}A{\hat{R}}_{i,t}, \end{array}$$

where *t* ∈ *w* = [*t*_2_, *t*_3_] and N is the total number of observations sample. Abnormal return and average abnormal return can be accumulated over time. Cumulative abnormal return (CAR) of index i is calculated over a period from t2 to t3, and cumulative average abnormal return (CAAR) is calculated based on the following equations:

(5) $$\begin{array}{c} {\text{CAR}}_{i,}\left(t_{2},t_{3}\right)=\sum_{t=t_{2}}^{t_{3}}AR_{i,t}, \end{array}$$

(6) $$\begin{array}{c} \text{CAAR}\left(t_{2},t_{3}\right)=\sum_{t=t_{2}}^{t_{3}}AAR_{t}. \end{array}$$

*(2) Significance Tests. After demonstrating the abnormal return, we plan to test these indices across four event windows, subindustries, asset scales, and firm ages with two nonparametric tests, namely the corresponding t-test (Boehmer, Musumeci and Paulson, 1991) and the GRANK test* [34]*, which are robust to event-induced volatility and cross-correlation of returns.*Therefore, it is calculated with the following equations (7) *and* (8),*respectively*:

(7) $$\begin{array}{c} t=\frac{\sum_{t=0}^{N}\left[\sum_{t_{1}}^{t_{2}}\left(AR_{i,t}/\hat{s}\right)/\sqrt{m}\right]}{\sqrt{N}}, \end{array}$$

where *m* represents the days in event window (*m* = *t*_2_ − t_1_ + 1), *t*_1_, *t*_2_ ∈ *w* = [*t*_2_, *t*_3_], and $\hat{s}$represents the variance of stock residuals in the estimation window.

Then,

(8) $$\begin{array}{c} t_{\text{grank}}=\frac{k_{0}-\left(1/2\right)}{S_{k}}, \end{array}$$

where $S_{k}=\sqrt{1/T\prime \sum_{t=T_{0}+1}^{T_{2}}n_{l}/n{\left({\bar{K}}_{l}-\left(1/2\right)\right)}^{2}}$ and ${\bar{K}}_{t}=\left(1/n_{l}\right)\sum_{i-1}^{n_{l}}K_{it}$.

## 4. Empirical Results

This paper selects the cumulative abnormal return (CAR) as the primary indicator to measure the short-term performance of the Malaysian stocks under the influence of lockdown announcements during the COVID-19 pandemic and calculates these statistics, namely the average abnormal return (AAR), cumulative average abnormal return (CAAR), and standard deviation for all sample companies within three days before and after the event. From the perspective of the whole sample and the subsample, we propose and demonstrate the impact of the four lockdown announcements on the market performance of the Malaysian healthcare industry.

### 4.1. Full-Sample Analysis

Events 1 to 4 indicate the announcements noted by the Malaysian government, such as 1st phase MCO of the event on March 16, 2020, 2nd phase MCO of the event on March 25, 2020, 3rd phase MCO of the event on April 10, 2020, and 4th phase MCO of the event on April 25, 2020, respectively.

Table 2 demonstrates the average abnormal return (AAR) surrounding the four lockdown events, and the first event had a more severe impact on the daily returns of 12 sample companies within three days before and after the event. The majority of average abnormal returns were negative and passed the significance test at the level of 1% (see Table 2). The duration of the second phase of MCO is less than ten days from the previous stages, and the influence of this announcement is not fully reflected in the stock market, leading to the results that the daily returns of sample companies shows an upturn at the begining of three trading days in event 1, and the abnormal return is showing a negatively related phenomenon. However, the sample companies' stock prices bounced back continuously, and the abnormal returns increased steadily. Furthermore, the following two events did not substantially impact the stock returns, and with the deregulation, the spanking of stock price slowed down.

To further unravel the story of the cumulative changes in daily returns within the event window, this research introduces CAR and CAAR to reflect the distribution of the CAR within sample companies and the change trajectory over time within three trading days before and after the event, shown in Table 3 and Figure 1, respectively.

Table 3 also presents the descriptive statistical results of CAAR under the impact of four events for the entire 12 sample companies (see Table 3). When the announcement occurred in the first phase, 9 of the 12 companies were negative, accounting for 75% of the sample companies. The returns of the most affected enterprises during the event window were as low as −37.6%, and the least affected sample had a maximum return of 8.8% for seven consecutive days. Moreover, referring to the average impact of the sample companies during the first phase of MCO, the overall CAAR of 12 samples is significantly negative, which indicates that each company's average cumulative abnormal loss has reached as high as 12.82% since the event.

As illustrated in Figure 1, the first phase of movement control announced by the Malaysian government not only had a significant negative impact on the stock performance of the healthcare industry but also influenced the stock prices of most companies negatively and more seriously (see Figure 1). Nevertheless, 11 of 12 companies have positive cumulative income within seven days before and after the introduction of the second phase of MCO. During this period, investors remained reluctant to invest due to concerns about the high degree of unpredictability and uncertainty in the stock market movements, including the healthcare stock. Since CAAR is the cumulative value of AAR, as shown in Table 3, within the second event, although the sample company's AAR is significantly negative (AAR = -0.0122) when the event window is −2, the sample companies contribute a positive CAAR at 9.38% (CAAR = 9.38%) and pass the 1% significant test. In this stage, the sample companies have effectively controlled the second movement control phase's impact. With the continuous deregulation in the following two phases, the impacts of the events on market performance also diminished and showed a steady rebound in the Malaysian healthcare industry.

In addition to the CAR cross-sectional data within the event window of (−3, 3), Figure 2 demonstrates the dynamic changes in CAAR within seven trading days (see Figure 2). The AAR performance of sample companies in the first phase is diametrically opposite to the following three phases, inducing that the fluctuation is more intuitively reflected in the CAAR in Figure 2 (see Figure 2). Concerning the response time of sample companies, the negative shock lasts longer than the positive one. The negative impact of the first movement control has been extended to another three trading days before the second phase of MCO.

With respect to the following three events, sample companies have rich experience in responding to the lockdown events, with a steady rebound under the precondition of stabilizing stock prices. Therefore, investors can approach the healthcare stock market more rationally, with more positive expectations for upcoming events, which also positively affect the market reaction significantly. As a highly demanded industry in a disease outbreak, demand factors are more critical than other disruptions in the Malaysian healthcare industry.

### 4.2. Subsample Analysis

#### 4.2.1. Subindustry

This article divides the company into three subindustries in which 12 healthcare companies are located Health Care Equipment & Services (0613, 516,7153, 7106, 7113), pharmaceuticals (7090, 7148, 7081, 7178), and healthcare providers (5225, 5878, 0101) considering.  Table 4 presents the magnitude of lockdown announcements' impact on companies' short-term performance in different subindustries (see Table 4). Referring to the first phase shows that the MCO regulation harms the short-term profitability of every subindustry. Meanwhile, the pharmaceutical industry has its most significant impact, followed by the industry of healthcare providers and then the Health Care Equipment & Services. In the following three phases, with the gradual relaxation of government regulation, the subindustry of Health Care Equipment & Services and Pharmaceuticals shows a trend of stable and favorable, while compared with former ones, the stock performance of the healthcare provider industry fluctuates slightly. The increased demand for medical devices can explain this during the COVID-19 crisis that has boosted the healthcare companies' revenue significantly after the first lockdown event. Since the fourth event is a gradual deregulation order and the stock market is rebounding, healthcare providers had a negative CAAR in the last event, as the IHH, CMC, and KJP companies had a slightly negative influence since the continuing lockdown announcement.

#### 4.2.2. Asset Scale

According to the scale of the total assets published on the latest annual report, 12 companies are divided into three groups: small (7090, 0613, 0101, 7178), medium (7148, 7153, 7081, 7106), and large (5168, 5225, 5878, 7113), with every four companies, respectively. The results in Table 5 support that lockdown events have different influences on stock returns according to firm sizes. These four events have an overall more negligible impact on large asset-scale companies, and the impact is relatively more prominent on medium-scale and small-scale companies (see Table 5). The first-phase event harms overall stock performance. With the deregulation of MCO, the impact changes from negative to positive, while the small-scale and medium-scale samples always bear the brunt. It also illustrates that the larger company with grander asset scale is related to less negative returns over the disease outbreak period.

On account of funds, experience, or coping strategies, healthcare companies with relatively more minor asset scales are at a disadvantage compared with the larger ones [16]. Overall, relatively smaller asset scale ones have greater risk exposure and are more powerless against the risks at the time of events.

#### 4.2.3. Firm Age

This article divides 12 healthcare companies into two groups by firm ages since the date of its initial public offering (IPO). The average age of whole sample is 17.04 years. When the firm age is below 17.04 years, this firm is assigned to the “young group” (0613, 5168, 5225, 0101, 7178); otherwise, it is assigned to the “old group” (7090, 7148, 7153, 5878, 7081, 7106, 7113).

Compared with younger firms, older firms are more affected by the lockdown events from the results shown in Table 6. Four events have significant impacts on the daily returns of the old group. However, Table 6 shows that within the young firms, only the CAAR under the third event shows statistical significance, which means the younger firms group impacts their stock returns during the third event. Furthermore, Table 6 supports that the impact of event 1 on an old firm group is more significant than that on a young one. This result suggests that the negative relationship between the stock market and lockdown is weaker for young firms. These findings are consistent with Tang et al. [35] on the Chinese market that older firms have more processes, entrenched routines, and social embeddedness. It means that the firms have greater inertia, making it harder to adjust or reposition in response to external developments [36]. In consequence, when faced with major environmental disruptions such as the global pandemic COVID-19, older companies encounter more problems than the young in routine activities of existing businesses in the context of the first strict lockdown, so the negative impact is more severe in event 1 (see Table 6).

### 4.3. Robustness Check

The significance of the coefficients changes slightly when the market model is changed to other market models, so the market adjusted model is taken into account in this paper. Not surprisingly, as shown in Table 7, we introduce CAR and CAAR to reflect the distribution of the CAR within sample companies and the change trajectory over time within three trading days before and after the event under the market adjusted model, and the significance of the coefficients is the same as the market model, which means the results of this paper are reliable.

## 5. Conclusion and Implication

### 5.1. Conclusion

This article examined the impact of four lockdown events on the stock returns of 12 listed healthcare companies in Malaysia by employing the event study methodology. The results support that lockdown events affect the short-term market performance of 12 healthcare companies listed in Bursa Malaysia. According to the strict movement control, event 1 has the most significant negative impact on samples. Nevertheless, the impacts of the subsequent three events decrease and become satisfactory around the event day. In line with uncertainty theory [31], investors became worried at the moments of uncertainly during the first lockdown announcement event, with the deregulation of movement control and the apparent effect of stopping the COVID-19 virus from spreading the first event, and as a highly demanded sector in disease, resulting in a rebound improvement in the performance of healthcare stocks. Therefore, the Malaysian, including stock investors, expected the government to impose a lockdown, as shown in the stock market's returns by the upcoming three lockdowns. Moreover, the lockdown events have different effects on healthcare firms regarding subindustry, firm ages, and asset scale. Firms that belong to the pharmaceutical subindustry are more impacted by the events than Health Care Equipment & Services and healthcare provider subindustries. Meanwhile, large-scale companies have an advantage over small-scale companies in coping strategies and capital reserves. Moreover, older firms are more affected by the events than younger companies, which have more flexible ways to reduce the negative impacts and stabilize the stock price [37].

### 5.2. Implication

The market reactions to the four MCO events are different. The first announcement of MCO is under more strict government regulation. Investors can overhaul their stock portfolios, choosing larger-scale but younger companies that belong to the healthcare industry to minimize the adverse effects of MCO considering the COVID-19 pandemic and, in the process of gradual deregulation, choosing subindustry that belongs to healthcare provider industry, whose market reaction is better than others. Although many countries have adopted similar measures to control the spread of the epidemic, these countries have also paid the price of painful economic stagnation or retrogression. In this regard, market participants are divided on whether the Malaysian government authorities will take this measure. Once the order of MCO on March 16, 2020, comes into effect, this panic spreads quickly to the whole stock market. Investors behaved irrationally, and the price of stocks fell dramatically. Investors' overreaction can be explained in the context of the lockdown order [38].

However, after the first MCO, the market participants gradually returned to normal with the following events. On the one hand, the stricter lockdown order causes an economic disruption and a negative shock on the stock performance generally. On the other hand, the demand for health care is increasing as the policy has released a signal of severe infection. Meanwhile, the expectation of strict lockdown order has been formed and stable among investors. Nevertheless, the stock price fluctuation also depends on the company's characteristics. The event effect is more pronounced in mature small healthcare companies, which belong to the pharmaceutical subindustry. Meanwhile, large-scale companies have an advantage over small-scale companies in coping strategies and capital reserves. Referring to the demand surge of medical items in disease outbreaks [12], the subsequent three extensions of MCOs have positively impacted the stock returns of healthcare companies in Malaysia. In the following events, the policy shock has less impact than the first announcement. The sample companies also have more experience in responding to lockdown orders and stabilizing stock prices. Last but not least, the spread of COVID-19 is partly controlled by the first lockdown order, somehow mitigating the negative impacts of pandemics. Before the MCO announcements, the market had even formed expectations, and the trading behavior returned to rationality. The investors regard the news of the lockdown positively and ultimately reflected on the stock return indices, and they can take steps before trading during the lockdown period, especially in the early phase of lockdown, to avoid the volatility of stocks. Furthermore, the stock market has positively affected the announcement of lockdown after the first event, and demand factors are more critical than other disruptions for the Malaysian healthcare sector.

This paper has several limitations, one of which is that since COVID-19 is still ongoing, we have only studied the short-term impact on the market reaction of listed Malaysia healthcare companies, excluding unlisted ones. Other events are happening during the pandemic, such as tax reduction policy and cut to interest rates, and these are also suggestions for future research. Another limitation is the slackness of data, and this paper did not study sociodemographic variables in terms of investors, such as age, gender, financial literacy, and stock market experience.

## Figures and Tables

**Figure 1:** Average abnormal return (AAR) changes over event window.

**Figure 2:** Cumulative average abnormal return (CAAR) changes over the event window.

**Table 1:** Distributions of 13 healthcare companies listed in Malaysia.

Stock code	Definition	Abbreviation	Age^1^	Asset scale (bill RM)^2^	Subindustry
7090	Apex Healthcare Berhad	AHEALTH	20	583.166	Pharmaceuticals
0163	Careplus Group Berhad	CAREPLS	9	272.080	Health Care Equipment & Services
7148	Duopharma Biotech Berhad	DPHARMA	18	919.801	Pharmaceuticals
5168	Hartalega Holdings Berhad	HARTA	12	3,317.582	Health Care Equipment & Services
5225	IHH Healthcare Berhad	IHH	8	45,053.289	Healthcare providers
7153	Kossan Rubber Industries Berhad	KOSSAN	24	2,355.142	Health Care Equipment & Services
5878	KPJ Healthcare Berhad	KPJ	25	5,985.847	Healthcare providers
7081	Pharmaniaga Berhad	PHARMA	20	1,592.302	Pharmaceuticals
7106	Supermax Corporation Berhad	SUPERMX	20	1,842.708	Health Care Equipment & Services
0101	TMC Life Science Berhad	TMCLIFE	14	848.516	Healthcare providers
7113	Top Glove Corporation BHD	TOPGLOV	19	5,688.205	Health Care Equipment & Services
7178	Y.S.P Southeast Asia Holding Berhad	YSPSAH	16	431.737	Pharmaceuticals

(2) The variable of firm age measures the years between the date of company's IPO and May 31, 2020.) The data of firm size come from company's latest balanced sheet, retrieved on May 25, 2020.

**Table 2:** Average abnormal return (AAR) over the event window.

Event window	Event 1	Event 2	Event 3	Event 4
−3	0.0003	0.0071	0.0109^*∗∗*^	−0.0037
	(0.073)	(0.975)	(2.147)	(−0.578)
−2	0.0068	−0.0122^*∗∗*^	−0.0063	−0.0222^*∗∗∗*^
	(1.434)	(−2.237)	(−1.329)	(−3.233)
−1	−0.0314^*∗∗∗*^	0.0302^*∗∗∗*^	0.0139^*∗∗∗*^	0.0262^*∗∗∗*^
	(−4.956)	(5.947)	(2.909)	(4.053)
0	−0.0572^*∗∗∗*^	0.0102^*∗∗*^	0.0023	0.0096
	(−9.477)	(1.989)	(0.473)	(1.485)
1	−0.0119^*∗∗*^	0.0206^*∗∗∗*^	0.0222^*∗∗∗*^	0.0305^*∗∗∗*^
	(−2.482)	(4.438)	(4.651)	(4.682)
2	−0.0141^*∗∗∗*^	0.0196^*∗∗∗*^	0.0068	0.0082
	(−3.028)	(4.139)	(1.407)	(1.269)
3	−0.0208^*∗∗∗*^	0.0184^*∗∗∗*^	0.0060	−0.0057
	(−4.402)	(3.912)	(1.224)	(−0.876)

(1) ^*∗*^Significant at the 10% level. ^*∗∗*^Significant at the 5% level. ^*∗∗∗*^Significant at the 1% level. *p* value denoted in parentheses.

**Table 3:** Statistical results on the full sample.

Event no.	Obs.	Coef.	*T*_grank_ value	Min	Max	Std. D	CAR>0	CAR<0
1	12	−0.1282^*∗∗*^	−2.473	−0.376	0.088	0.145	3	9
2	12	0.0938^*∗∗∗*^	3.393	−0.104	0.278	0.097	11	1
3	12	0.0556^*∗∗∗*^	3.687	−0.005	0.111	0.039	11	1
4	12	0.0428	0.777	−0.016	0.188	0.069	8	4

^*∗*^Significant at the 10% level. ^*∗∗*^ Significant at the 5% level. ^*∗∗∗*^Significant at the 1% level.

**Table 4:** Cumulative abnormal average return (CAAR) in 3 subindustries.

Event no.	Subindustry					
	Health Care Equipment & Services		Pharmaceuticals		Healthcare providers	
	CAAR	*T*_grank_ value	CAAR	*T*_grank_ value	CAAR	*T*_grank_ value
1	−0.0666	−0.327	−0.2394^*∗∗∗*^	−3.422	−0.0831	−1.139
2	0.1122^*∗∗∗*^	2.848	0.1270^*∗∗∗*^	3.429	0.0192	−0.330
3	0.0723^*∗∗∗*^	3.285	0.0531^*∗∗*^	3.215	0.0314	0.419
4	0.0806	0.673	0.0326	1.475	−0.0066	−0.965

^*∗*^Significant at the 10% level. ^*∗∗*^Significant at the 5% level. ^*∗∗∗*^Significant at the 1% level.

**Table 5:** Cumulative abnormal average return (CAAR) in 3 sample scales.

Event no.	Sample scale					
	Small		Medium		Large	
	CAAR	*T*_grank_ value	CAAR	*T*_grank_ value	CAAR	*T*_grank_ value
1	−0.2099^*∗∗∗*^	−3.299	−0.1847^*∗∗∗*^	−3.034	0.0097	0.995
2	0.1352^*∗*^	1.780	0.1207^*∗∗∗*^	3.225	0.0256	0.647
3	0.0682^*∗∗∗*^	2.712	0.0789^*∗∗∗*^	3.307	0.0199	0.496
4	0.0578	1.556	0.0584	0.150	0.0122	0.089

^*∗*^Significant at the 10% level. ^*∗∗*^Significant at the 5% level. ^*∗∗∗*^Significant at the 1% level.

**Table 6:** Cumulative abnormal average return (CAAR) in 2 sample ages.

Event no.	Firm age			
	Young group		Old group	
	CAAR	*T*_grank_ value	CAAR	*T*_grank_ value
1	−0.1019	−0.939	−0.1471^*∗∗*^	−2.536
2	0.0709	0.809	0.1102^*∗∗∗*^	4.015
3	0.0529^*∗∗*^	0.809	0.0577^*∗∗∗*^	2.908
4	0.0416	0.362	0.0437	0.758

^^*∗*^^^Significant at the 10% level.^^ ^*∗*^ ^*∗*^^^Significant at the 5% level.^^ ^*∗*^ ^*∗*^ ^*∗*^^^Significant at the 1% level.^

**Table 7:** Cumulative average abnormal return (CAAR) over event window with two models.

Items	Market model				Market adjusted model			
	Event 1	Event 2	Event 3	Event 4	Event 1	Event 2	Event 3	Event 4
Coef.	−0.1282^*∗∗*^	0.0938^*∗∗∗*^	0.0556^*∗∗∗*^	0.0428	−0.1185^*∗∗*^	0.0988^*∗∗∗*^	0.0568^*∗∗∗*^	0.0438
*T*_grank_	−2.473	3.393	3.687	0.777	−2.419	3.341	3.584	0.809
CAR>0	3	11	11	8	3	11	11	8
CAR<0	9	1	1	4	9	1	1	4
Obs.	12	12	12	12	12	12	12	12

^^*∗*^^^Significant at the 10% level.^^ ^*∗*^ ^*∗*^^^Significant at the 5% level.^^ ^*∗*^ ^*∗*^ ^*∗*^^^Significant at the 1% level.^

## Data Availability

The sample data selected in this article are listed healthcare industry companies in Bursa Malaysia. The database we used for this study is FTSE Bursa Malaysia KLCI (FBMKLCI).
